# The Potential Therapeutic Role of Exosomal MicroRNA-520b Derived from Normal Fibroblasts in Pancreatic Cancer

**DOI:** 10.1016/j.omtn.2019.12.029

**Published:** 2020-01-10

**Authors:** Huijuan Shi, Hui Li, Tiantian Zhen, Yu Dong, Xiaojuan Pei, Xiangliang Zhang

**Affiliations:** 1 Department of Pathology, The First Affiliated Hospital of Sun Yat-sen University, Guangzhou 510080, P.R. China; 2 Department of Pathology, Shenzhen Hospital of Southern Medical University, Shenzhen 518110, P.R. China; 3 Affiliated Cancer Hospital and Institute of Guangzhou Medical University, Guangzhou 510095, P.R. China

**Keywords:** exosomes, microRNA-520b, fibroblasts, pancreatic cancer, ZNF367

## Abstract

Pancreatic cancer (PC) remains a major health concern, with conventional cancer treatments exerting little influence on the disease course. MicroRNA-520b (miR-520b) functions as a tumor suppressor in several types of human cancers, whereas its anti-tumor property in the context of PC is still fundamental. The aim of this study is to identify the potential therapeutic role of miR-520b, transferred by exosomes, derived from normal fibroblasts (NFs) in PC progression. A gain-of-function study was performed to examine the roles of miR-520b in PC cell line SW1990, which suggested that miR-520b served as a tumor suppressor in PC. In order to confirm the role of exosomal miR-520b, exosomes were isolated from NF culture medium and cocultured with SW1990 cells. During the coculture experiments, we disrupted exosome secretion and upregulated exosomal miR-520b. The *in vitro* coculture studies revealed that miR-520b was transferred from NF-derived exosomes to PC cells and thereby suppressed PC cell proliferation, invasion, migration, and stimulated apoptosis. Furthermore, inhibited tumor growth and live metastasis upon elevated miR-520b in exosomes were observed *in vivo*. Conjointly, our study demonstrates that NF-derived exosomal miR-520b impedes the progression of PC, which contributes to a novel, therapeutic role of exosomal miR-520b for treating PC.

## Introduction

Pancreatic cancer (PC) is an extremely aggressive malignancy with an alarmingly high incidence and high mortality rates.^1^^,^^2^ An existing study documented the deaths of 5,550 patients among the 6,220 newly diagnosed cases of PC patients in China in 2009.^3^ The associated risk factors of PC involve family history, chronic or hereditary pancreatitis, intraductal mucin-producing neoplasm, deficiency of vitamin D, high body mass index, and unhealthy life habits.^4^^,^^5^ Surgical resection is the only curative intervention for patients suffering from PC, with compliance in less than 15% of PC patients.^6^ Despite the advances, a poor prognosis is persistent in unresectable cases because of distant metastases or the local advancement, resulting in significant mortality among PC patients.^7^ Therefore, the development of new therapeutic modalities is essential for PC treatment.

MicroRNAs (miRNAs) are endogenous noncoding RNAs with varying lengths of approximately 23 nt, which exhibit vital functionality in post-transcriptional-repressive regulatory processes in plants and animals by binding to respective protein-coding genes.^8^ As a member of the miRNA family, miR-520b precedes its functionality along the progression of tumors in different types of cancers.^9^^,^^10^ For instance, the miR-520/373 family exerts its anti-metastasis properties in breast cancer by suppressing the secretion and expression of various proinflammatory cytokines.^11^ Moreover, miR-520b was found to exercise an inhibitory effect on cellular proliferation, invasion, and migration in spinal osteosarcoma.^12^

Exosomes are tiny membrane vesicles of endocytic nature secreted from a variety of cell types, which are regarded as key mediators in intercellular communications.^13^ A previous *in vivo* experiment has flagged the potential of exosomes hailed from human bone marrow mesenchymal stem cells to accelerate tumor growth.^14^ Furthermore, studies have reported the ability of exosomes to serve as promising vectors carrying lipid mediators, miRNAs, and various types of proteins.^15^ An existing study reported the presence of certain kinds of miRNAs in tumor-derived exosomes; for instance, exosome-derived miR-302b is involved in regulating proliferation in lung cancer cells.^16^

Therefore, we investigated whether exosomal miR-520b, derived from normal fibroblasts (NFs), could be transferred into PC cells so as to insinuate a potential regulatory role of exosomal miR-520b with respect to PC. In this study, zinc finger protein 367 (ZNF367) was predicted to be a target of miR-520b based on the predictions from the miRDB, microRNA.org, miRWalk, and starBase v2.0 databases. ZNF367 is a member of the ZNF family, which is found to be overexpressed in adrenocortical carcinoma, malignant pheochromocytoma/paraganglioma, and thyroid cancer.^17^ Hence, this study was designed to investigate the potential function of exosomal miR-520b in PC via regulation of ZNF367.

## Results

### The miR-520b Is Downregulated in PC

First, to screen for PC-related miRNAs, the microarray Gene Expression Omnibus (GEO): GSE50632 was analyzed by bioinformatics prediction. The low expression of miR-520b in serum of PC patients (Figure 1A) and in serum-derived PC exosomes was witnessed (Figure 1B). Quantitative reverse transcriptase polymerase chain reaction (qRT-PCR) was conducted for determining miR-520b expression in 6 PC cell lines (SW1990, Capan-1, AsPC-1, MIAPaCa-2, PANC-1, and PC-3). The results showed that miR-520b was downregulated in all 6 PC cell lines in comparison to the human pancreatic cell line HPC-Y5 (Figure 1C). As miR-520b exhibited the lowest expression in SW1990 cells among the 6 PC cell lines (p < 0.05), the SW1990 cell line was selected for further experiments.

**Figure 1:** Low Expression of miR-520b Is Observed in PC (A and B) The heatmap of differentially expressed miRNAs in the PC serum sample from GEO: GSE50632 (A) and the heatmap of key miRNAs in exosomes from GEO: GSE50632 (B) (the x axis represented the sample number; the y axis represented the name of differentially expressed miRNAs). The histogram in the upper right was the color gradation, with the changed color from top to bottom in which each of the rectangles corresponds with an expression pattern value of a sample, and each line showed the expression pattern of all genes. The dendrogram in the left displayed the cluster analysis results of differentially expressed miRNAs from different samples. The top bar showed the sample type. In the upper-right color gradation, blue represented normal control sample, and red displayed the tumor sample. (C) qRT-PCR showed that the lowest expression pattern of miR-520b was observed in SW1990 among 6 examined PC cell lines (SW1990, Capan-1, AsPC-1, MIAPaCa-2, PANC-1, and PC-3) relative to HPC-Y5 cells. *p < 0.05 versus HPC-Y5. Data in the figure were measurement data, which were expressed as mean ± standard deviation and compared by one-way ANOVA; the experiment was repeated 3 times independently.

### Ectopic Expression of miR-520b or Coculture with NFs Inhibits PC Cell Proliferation, Migration, and Invasion and Induces Apoptosis

To investigate the influence of miR-520b on the biological function of PC cells, cell proliferation, migration, invasion, and apoptosis were assessed after introduction of the miR-520b mimic into the SW1990 cells. The results in Figures 2A–2D displayed decreased proliferation, migration, and invasion in SW1990 cells transfected with the miR-520b mimic, with increased cell apoptosis compared to the SW1990 cells transfected with the mimic-negative control (NC; p < 0.05). These results suggested that the overexpression of miR-520b could inhibit the proliferation, migration, and invasion, whereas accelerate the apoptosis of PC cells.

**Figure 2:** miR-520b Overexpression Inhibits PC Cell Proliferation, Migration, and Invasion yet Promotes Apoptosis (A) miR-520b mimic inhibited SW1990 cell proliferation detected by the EdU assay. (B) miR-520b mimic promoted SW1990 cell apoptosis detected by flow cytometry. (C) miR-520b mimic inhibited SW1990 cell migration by the Transwell assay (×200). (D) miR-520b mimic suppressed SW1990 cell line invasion by the Transwell assay (×200). (E) miR-520b mimic in the NFs inhibited the proliferation of PC cells detected by the EdU assay. (F) miR-520b mimic in the NFs promoted PC cell apoptosis detected by flow cytometry. (G) miR-520b mimic in the NFs suppressed the migration of PC cells detected by the Transwell assay (×200). (H) miR-520b mimic in NFs disrupted the invasion of PC cells detected by the Transwell assay (×200). Data in the figure were presented as mean ± standard deviation, and the difference of which between two groups was compared by independent-sample t test. The experiment was repeated 3 times independently.

Since miR-520b was predicted with a lowered expression in PC, NFs transfected with the miR-520b mimic were cocultured with SW1990 cells to investigate whether NFs overexpressing miR-520b would affect the biological functions of PC cells. The PC cell proliferation, apoptosis, migration, and invasion were monitored. As shown in Figures 2E–2H, PC cells, cocultured with miR-520b mimic-transfected NFs, exhibited significantly decreased proliferation, migration, and invasion ability but a significantly increased cell apoptosis rate (p < 0.05). These results show that the coculture of NFs could influence the biological functions of PC cells.

### Disruption of Exosome Secretion in NFs Promotes PC Cell Invasion and Migration

To study whether miR-520b could be transfected into PC cells by exosomes *in vitro*, an exosome inhibitor GW4869 was employed in the NFs/PC coculture system, and the exosome release and miR-520b expression were documented. According to the acetylcholinesterase activity-detection results (Figure 3A), the cocultured cells exhibited significantly decreased acetylcholinesterase activity after GW4869 treatment, which denoted a decline in exosomes release. The results of the biological function investigation of NFs/PC coculture cells, with or without GW4869 treatment, revealed that the migration and invasion abilities of PC cells in NFs/PC coculture system increased significantly, but miR-520b expression was reduced after GW4869 treatment (p < 0.05; Figures 3B–3F). The aforementioned findings suggest that GW4869, the inhibitor of exosomes, may suppress the miR-520b expression by inhibiting the release of exosomes. This reduced exosome release can influence the biological functions of PC cells.

**Figure 3:** The Migration and Invasion of PC Cells Are Promoted by Suppressing the Release of Exosomes (A) The release of exosomes after GW4869 treatment in the coculture system of SW1990 cells and NFs by acetylcholinesterase activity detection. (B) Representative images of migration ability of SW1990 cells cocultured with NFs after GW4869 treatment assessed by the Transwell assay (×200). (C) The migration rate of SW1990 cells cocultured with NFs after GW4869 treatment assessed by the Transwell assay. (D) miR-520b expression after GW4869 treatment in SW1990 cells cocultured with NFs determined by qRT-PCR. (E) Representative images of the invasion ability of SW1990 cells cocultured with NFs after GW4869 treatment detected by the Transwell assay (×200). (F) The invasion rates of SW1990 cells cocultured with NFs after GW4869 treatment detected by the Transwell assay. PC, pancreatic cancer. *p < 0.05 versus the coculture + DMSO group. Data in the figure were measurement data, which were presented as mean ± standard deviation, and the difference of which between two groups was compared by independent-sample t test. The experiment was repeated 3 times independently.

### NFs Secrete miR-520b-Containing Exosomes

In order to investigate the transfer of miR-520b expression from the exosomes to PC cells, the isolated extracellular vesicles were observed under transmission electron microscope (TEM), and the miR-520b expression was determined by performing qRT-PCR. The NF-secreted exosomes are characterized with different sizes and a sphere structure enveloped by a lipid bilayer membrane (Figure 4A). The external surface of NF-derived exosomes was manifested with a deeply dyed area of the bilayer lipid molecular membrane, whereas the internal surface was evident with a superficially dyed area of heterogeneity, and the partial substance with the density of protein was visible (Figure 4A). As detected using a nanoparticle tracking analyzer, the isolated microvesicle samples presented with an average size of 100 nm (Figure 4B). Subsequently, the western blot analysis confirmed that the isolated extracellular vesicles were positive for exosome markers CD63, Alix, and TSG101 but negative for calnexin (Figure 4C). Conjointly, these results ascertained the release of NF-secreted exosomes. To examine the presence of miR-520b in NF-derived exosomes, miR-520b mimic was introduced into NFs, and the qRT-PCR results revealed an elevated miR-520b expression in exosomes derived from NFs transfected with miR-520b mimic (Figure 4D). The aforementioned data indicate the ability of NFs to release exosomes carrying miR-520b.

**Figure 4:** Exosomes Containing miR-520b Could Be Produced by NFs (A) The ultrastructure of exosomes produced by NFs observed under the TEM (×5,000). (B) The size-distribution profile of exosomes by nanoparticle tracking analysis. (C) The expression of exosome markers CD63, Alix, TSG101, and negative marker calnexin, confirmed by western blot analysis. (D) miR-520b expression in the exosomes determined by qRT-PCR. Data in the figure were analyzed by independent-sample t test. The experiment was repeated 3 times independently.

### NF-Derived Exosome Internalization in PC Cells

In order to investigate the relationship between PC cells and miR-520b in the NF-derived exosomes, the exosomes in NFs with PKH26 were labeled and cocultured with SW1990 cells. After a 6-h regimen of coculture, little red fluorescence was evident in the SW1990 cells, which revealed the penetration of few PKH26-labeled exosomes into the SW1990 cells. After a 12-h regimen of coculture, red fluorescence was observable in a small amount of SW1990 cells, with key fluorescence concentration in the cytoplasm. These results indicated that the PKH26-labeled exosomes were predominantly located in the cytoplasm of SW1990 cells after internalization. Evident red fluorescence was reflective in an increasing number of SW1990 cells upon extending the time of coculture, which indicated that the number of PKH26-labeled exosomes internalized by SW1990 cells increased in a time-dependent manner. After a 48-h regimen of coculture, the PKH26-labeled exosomes were evident in SW1990 cells (Figure 5).

**Figure 5:** The Exosomes from NFs into SW1990 Cells Increased in a Time-Dependent Manner (×400) SW1990 cells were cocultured with PKH26-labeled exosomes (red). SW1990 cells were stained with FITC-conjugated phalloidin (green) and nuclei stained with DAPI (blue). The experiment was repeated 3 times independently.

### Ectopic Expression of Exosomal miR-520b Inhibits PC Cell Proliferation, Migration, and Invasion and Induces Apoptosis

In order to study whether exosomal miR-520b could influence the biological function of PC cells, the proliferation, migration, invasion, and apoptosis of SW1990 cells were assessed upon exosomal miR-520b upregulation by coculture with exosomes from NFs overexpressing miR-520b. The results in Figures 6A–6H showed that compared to the Exo-miR-NSM group, the Exo-miR-520b group exhibited significantly diminished proliferation, migration, and invasion ability but a notably increased apoptosis rate (p < 0.05). Furthermore, the results of western blot analysis (Figures 6I and 6J) demonstrated that compared to the Exo-miR-NSM group, the Exo-miR-520b group had remarkably decreased expression of several proliferation-related proteins (Ki67 and proliferating cell nuclear antigen [PCNA]), invasion-related proteins matrix metalloprotein (MMP)-2 and MMP-9 (p < 0.05). The aforementioned results indicated that PC cell proliferation, migration, and invasion are inhibited, whereas cell apoptosis is stimulated by overexpression of miR-520 in exosomes.

**Figure 6:** Exosomal miR-520 Overexpression Derived from NFs Inhibits Proliferation, Migration, and Invasion and Promotes Apoptosis of PC Cells (A) Representative images of proliferation of SW1990 cells in a coculture system with exosomes derived from NFs detected by the EdU assay (×200). (B) Proliferation rate of SW1990 cells was suppressed by miR-520b in the exosomes derived from NFs. (C) miR-520b in the exosomes derived from NFs increased SW1990 cell apoptosis revealed by flow cytometry. (D) Apoptosis rate of SW1990 cells was enhanced by miR-520b in exosomes derived from NFs. (E) Representative images of SW1990 cell migration ability in a c-culture system with exosomes derived from NFs demonstrated by the Transwell assay (×200). (F) Migration rate of SW1990 cells was decreased by miR-520b in exosomes derived from NFs. (G) Representative images of SW1990 cell-invasion ability in a coculture system with exosomes derived from NFs revealed by the Transwell assay (×200). (H) Invasion of SW1990 cells was decreased by miR-520b in the exosomes derived from NFs. (I) Protein band diagram of proliferative markers (Ki67, PCNA) and invasive markers(MMP-2, MMP-9) in exosomes derived from NFs detected by Western blot analysis. (J) Expression of proliferative markers (Ki67, PCNA) and invasive markers (MMP-2, MMP-9) in exosomes derived from NFs determined by Western blot analysis.. *p < 0.05 versus the Exo-miR-NSM group. Data in the figure were denoted as measurement data, which were expressed as mean ± standard deviation, and the difference of which between two groups was compared by independent-sample t test. The experiment was repeated 3 times independently.

### miR-520b Targets and Negatively Regulates ZNF367 in PC Cells

To identify the target genes of miR-520b, a combination of mRNA-miRNA interaction prediction was conducted using databases miRDB (http://www.mirdb.org/), microRNA.org (http://34.236.212.39/microrna/getMirnaForm.do), miRWalk (http://mirwalk.umm.uni-heidelberg.de/), and starBase v2.0 (). POLK, GALNT3, ZNF367, and TGFBR2 were predicted as potential target genes of miR-520b (Figure 7A). The heatmap of GEO: GSE71989 displayed that ZNF367 was highly expressed in PC (Figure 7B), whereas other genes were not differentially expressed in PC-related microarray data. Besides, TargetScan highlighted the presence of a binding region between miR-520b and ZNF367. In order to ascertain the presence of binding sites between miR-520b and ZNF367 and whether ZNF367 was a direct target gene of miR-520b, a dual-luciferase reporter gene assay was conducted. On that basis, the data of the dual-luciferase reporter gene assay, shown in Figure 7C, exhibited that the miR-520b mimic decreased luciferase activity after cotransfection with the ZNF367 wild type (ZNF367-WT), with insignificant alterations in the luciferase activity after cotransfection with the ZNF367 mutant (ZNF367-Mut) (p > 0.05). These results suggest that miR-520b can target the ZNF367 gene.

**Figure 7:** ZNF367 Is Targeted by miR-520b, and the Silencing of ZNF367 Inhibited PC Cell Proliferation, Migration, and Invasion (A) miRDB, microRNA.org, miRWalk, and starBase v2.0 databases were applied to predict the target genes of miR-520b. (B) The heatmap of differentially expressed genes in GEO: GSE71989 (the x axis represented sample number; the y axis represented the names of differential expressed genes). The histogram in the upper right represented color gradation with the change of color from top to bottom, which illustrated that the expression in the profiling data was in descending order. Each of the rectangles corresponded to the expression of each sample, and each column represented the expression of all genes. The dendrogram in the left was the cluster analysis results of different genes from different samples. The upper band represented the sample type. In the upper-right color gradation, blue represented the normal control sample, and red represented PC tumor sample. (C) Verification of the binding relationship between miR-520b and ZNF367 by the dual-luciferase reporter gene assay. (D) mRNA expression of differentially expressed genes in the PC cells determined by qRT-PCR. (E) Silencing of ZNF367 suppressed the proliferation of PC cells detected by the EdU assay (×200). (F) Silencing of ZNF367 enhanced the apoptosis of the PC cell detected by flow cytometry. (G) Silencing of ZNF367 suppressed the migration of PC cells detected by the Transwell assay (×200). (H) Silencing of ZNF367 decreased the invasion of PC cells detected by the Transwell assay (×200). *p < 0.05 versus the ZNF-367-Mut group. Data in the figure were measurement data, which were expressed as mean ± standard deviation and compared by independent-sample t test. The data of expression detected by qRT-PCR were compared by one-way ANOVA. The experiment was repeated 3 times independently.

qRT-PCR was conducted to determine the expression of POLK, GALNT3, ZNF367, and TGFBR2 in PC cells. ZNF367 expression was elevated in PC cells with the largest alterations among the above-mentioned genes (p < 0.05; Figure 7D). For further investigation, ZNF367 was knocked down with small interfering (si)RNA against ZNF367 to observe its influence on the proliferation, migration, invasion, and apoptosis of PC cells. Results showed that cell proliferation, migration, and invasion progressively decreased, but cell apoptosis increased after transfection with the siRNA targeting ZNF367 (si-ZNF367; p < 0.05; Figures 7E–7H). Therefore, we can conclude that ZNF367 depletion can inhibit the proliferation, migration, and invasion of PC cells, while simultaneously stimulating cell apoptosis.

### Upregulation of Exosomal miR-520b Reduces Tumor Growth and Liver Metastases

A tumor formation assay in nude mice was conducted in order to manifest the influence of exosomal miR-520b on PC growth. Results (Figures 8A–8C) showed that compared to the Exo-miR-NSM group, the Exo-miR-520b group, with increased miR-520b expression, showed lower tumor growth and a smaller-sized tumor (p < 0.05). Immunofluorescence staining consistently displayed decreased expression of invasion-related proteins (MMP-2 and MMP-9) in tumor tissues in the Exo-miR-520b group compared to the Exo-miR-NSM group (p < 0.05; Figure 8D). Meanwhile, hematoxylin and eosin (H&E) staining was conducted for observation of lymph node metastases after treatment with exosomes containing miR-520b. As displayed in Figures 8E–8G, the mice exhibited tumor metastasis of varying degrees. The tumor metastasis was repressed with a significantly decreased number of lymph metastatic nodes in the Exo-miR-520b group in comparison to the Exo-miR-NSM group (p < 0.05). Collectively, the aforementioned results suggested that the overexpression of exosomal miR-520b, derived from NFs, could suppress the tumor formation and metastasis.

**Figure 8:** Exosomal miR-520 Overexpression Inhibits Tumor Growth and Metastasis (A) The tumor volume of the PC tumor was inhibited after treatment with the exosomic miR-520b mimic. (B) Representative images of tumors formed in nude mice. (C) Detection of miR-520 expression by qRT-PCR. (D) Expression of invasive markers (MMP-2 and MMP-9) detected by immunofluorescence assay (×400). (E) Pictures of hepatic lymph node metastasis of nude mice after an 8-week injection with the transfected PC cell line SW1990 through the caudal vein (F) Liver morphology of nude mice after an 8-week injection with the transfected PC cell line SW1990 through the caudal vein. (G) The number of lymph metastatic nodes in nude mouse livers counted by H&E staining after injection with transfected PC cell line SW1990 for 8 weeks. *p < 0.05 versus the Exo-miR-NSM group. Data in the figure were measurement data, which were expressed as mean ± standard deviation and compared by independent-sample t test, n = 12.

## Discussion

In the research of miRNAs, hsa-miR-520h has been found to be involved in the inhibition of migration, invasion, and side populations of PC cells.^18^ Exosomes secreted from diverse cells are potential vectors transporting lipid mediators, miRNAs, and proteins, thereby functioning as extensive regulators of the intercellular communication and potential sources for drug release and gene therapeutic methods.^19^ The results from our study unraveled that miR-520b in exosomes produced by NFs could impede PC cell proliferation, migration, and invasion by negatively regulating ZNF367, which provided a promising therapy for PC patients.

Primarily, miR-520b was identified to be downregulated in patients suffering from PC. miR-520b, a member of miRNA family, was downregulated in LO2-X-S cells and clinical human hepatocellular carcinoma tissues.^20^ The key tumor-suppressive role of miR-520b has been implicated in a variety of human cancers.^21^^,^^22^ miRNAs are involved in tumorigenesis due to their regulatory functionality for downstream genes related to cancers after RNA transcription.^23^ miR-520c could impede the migration and invasion of glioma cells upon suppression of transforming growth factor-β receptor type 2, thus obstructing tumor cell growth and migration.^24^ Moreover, miR-520b could serve as a suppressant of cell growth, proliferation, invasion, and migration and promote the apoptosis of colorectal cancer cells by its inhibitory property in defective in cullin neddylation 1 domain containing 1.^22^ To conclude, the reduced expression of miR-520b could contribute to PC progression, whereas the upregulation of miR-520b could inhibit PC cell progression. Previously, upregulated exosomal miR-23b-3p has been proposed as a therapeutic target for the treatment of PC.^25^ In accordance with this finding, the results in our study presented that upregulated miR-520b in the exosomes derived from NFs inhibited the proliferation, migration, and invasion of PC cells, along with stimulation of PC cell apoptosis. An existing report has revealed the mutual interaction between PC cells and the NFs, which induces tumor cell invasion by coculture *in vitro* coculture.^26^ The successful coculture of PC cells and NFs in our study facilitated miR-520b to modulate cellular proliferation and apoptosis of PC cells. The *in vivo* experiment further supported the speculation that the overexpression of exosomal miR-520b, derived from NFs, could suppress the metastasis of PC cells and inhibit tumor formation.

Another significant finding is that miR-520b may target ZNF367, which was overexpressed in PC cells, the downregulation of which could inhibit proliferation, migration, and invasion and promote the apoptosis of PC cells. As serving as one of the tissue-specific transcription factors, ZNF367, when dysregulated, could disorder lipid development, metabolism, cell proliferation, adhesion, metastasis, and the differentiation processes.^27^ ZNF367 was reported as a direct target of miR-195, thus, extensively inhibiting tumor cell proliferation and promoting apoptosis.^17^ Furthermore, the knockdown of ZNF281, which is an alternative member of the zinc finger protein family, was identified to lower the overall survival of PC cells and function as an independent prognosis factor of PC.^28^ The aforementioned findings implied that upregulated miR-520b in NF-derived exosomes suppressed PC cell invasion and migration via downregulation of ZNF367.

To conclude, our key findings revealed that miR-520b was poorly expressed in PC. The upregulation of miR-520b in NF-derived exosomes may impede PC cell proliferation, migration, and invasion and induce apoptosis by targeting ZNF367 (Figure S1). In addition, these regulatory effects were verified by an *in vivo* assay as well. Based on these findings, miR-520b overexpression and silencing ZNF367 could serve as potential therapeutic targets for developing new therapeutic options for the treatment of PC.

## Materials and Methods

### Ethics Statement

The animal experiments were carried out with the approval of The First Affiliated Hospital of Sun Yat-sen University in accordance with the Guidelines for the Ethical Treatment of Animals. The least number of animals was included in the study, and animals were treated under the principle to reduce their pain.

### *In Silico* Analysis

The microarray data relevant to PC-derived exosomes were downloaded from the GEO database (https://www.ncbi.nlm.nih.gov/geo/). The limma package of R language was applied to screen out the differential gene expression in PC, with |log fold change| >2, a p value <0.05 as the threshold. A heatmap of differentially expressed miRNAs was retrieved using the pheatmap package array of R language. Next, the target genes of miR-520b were predicted using several databases, including miRDB (http://www.mirdb.org/), microRNA.org (http://www.microrna.org/microrna/microrna/getMirnaForm.do), miRWalk (http://mirwalk.umm.uni-heidelberg.de/), and starBase v2.0 (http://starbase.sysu.edu.cn/starbase2/index.php).

### Cell Selection

PC cell lines (SW1990, Capan-1, AsPC-1, MIAPaCa-2, PANC-1, and PC-3) and the human pancreatic cell line (HPC-Y5) were purchased from Yanhui Biotechnology (Shanghai, China) and cultured using Roswell Park Memorial Institute (RPMI)-1640 medium (SP1355; Shifeng Biological Technology, Shanghai, China) containing a combination of 10% fetal bovine serum (FBS), 100 U/mL penicillin, and 100 mg/mL streptomycin in a 5% CO_2_ incubator at 37°C. The medium was replaced every 1∼2 days. Upon attaining 80%∼90% cell confluence, the cells were subcultured. Lastly, qRT-PCR was performed to select the cell lines with the differentially expressed miR-520b.

### Culture of Primary NFs

NFs were extracted from the pancreatic tissues of 10-week-old wild-type C57 mice (Lianke Meixun Biomedicial Technology, Hangzhou, Zhejiang, China). Fresh pancreatic tissues were rinsed using D-Hanks solution, incised into pieces of 2∼3 cm^2^, and treated using collagenase at 37°C for 20 min, which was terminated by the addition of 10% Dulbecco’s modified Eagle’s medium (DMEM). The tissue sections were centrifuged at 1,000 *g* for 5 min, and the precipitate was resuspended and cultured in DMEM containing 15% FBS and 1% penicillin/streptomycin in a 5% CO_2_ incubator at 37°C. NFs were selected using the differential adhesion method, and the NFs at passages 2–5 were used for subsequent experiments.

### Cell Transfection

si-ZNF367 and NC siRNA (si-NC) were purchased from Santa Cruz Biotechnology (Santa Cruz, CA, USA), and miRNA-520b mimic, mimic-NC, miRNA-520b inhibitor, and inhibitor NC were from Shanghai GenePharma (Shanghai, China). NFs and SW1990 cells were transfected with above-mentioned plasmids or sequences using Lipofectamine 2000 (Invitrogen, Carlsbad, CA, USA). Following 48 h transfection, qRT-PCR was performed to assess transfection efficiency.

### Coculture of PC Cells and NFs

PC cell line SW1990 and NFs were treated using trypsin, centrifuged at 1,000 *g* for 5 min, and resuspended in 3 mL DMEM. The suspension (1 mL) was diluted 20 times, 10 μL of which was subjected onto a cell-count plate for cell counting. Afterward, the SW1990 and NFs were cocultured in a coculture chamber with a 4-μm porous membrane in the ratio of 3:1. The SW1990 cells (1.2 × 10^5^) were seeded in the apical chamber and cultured using DMEM containing 10% serum. The NFs (0.4 × 10^5^) were then seeded in a basolateral chamber and cultured using DMEM containing 15% serum. SW1990 cells and NF cells were cocultured under the aforementioned conditions for 4∼5 days, with medium replacement every 1∼2 days. The medium in the apical and basolateral chambers was renewed simultaneously. After coculture, the apical chamber was removed, and the cells were collected for further experiments.

### Dual-Luciferase Reporter Gene Assay

Primarily, the 3′ untranslated region fragment of ZNF367 was synthesized, which was then transfected into the pMIR-reporter plasmids (Huayueyang Biotechnology, Beijing, China) via the endonuclease sites SpelI and HindIII. The Mut sites of the complementary sequence on the ZNF367-WT plasmid were designed. After cleavage using restriction endonuclease, the target fragment was inserted into the pMIR-reporter plasmids using T4 DNA ligase. The WT and Mut plasmids (ZNF367-WT and ZNF367-Mut) with the correct sequences were separately cotransfected with miR-520b into the HEK293T cells (Beinuo Biotechnology, Shanghai, China). After transfection for 48 h, the cells were collected and lysed, followed by assessment of the luciferase activity using a dual-luciferase assay kit (K801-200; BioVision Technologies, Exton, PA, USA) on a GloMax 20/20 luminometer (Promega, Madison, WI, USA).

### qRT-PCR

TRIzol reagent (Invitrogen, Carlsbad, CA, USA) was added to extract the total RNA from cells in each group. After determination of the RNA concentration with a NanoDrop 2000 (Thermo Fisher Scientific, Waltham, MA, USA), 1 μg total RNA was transcribed into cDNA using a PrimeScript RT reagent kit in combination with the gDNA Eraser kit (Takara, Tokyo, Japan). After addition of 5 × DNA Eraser buffer and gDNA Eraser for genomic DNA termination at 42°C for 2 min, the cDNA was synthesized by a reaction at 37°C for 15 min and 85°C for 5 s. The quantitative real-time PCR was performed using a SYBR *Premix Ex Taq* (Tli RNaseH Plus) kit (Takara, Tokyo, Japan) on the quantitative real-time PCR instrument (ABI7500; Thermo Fisher Scientific, Waltham, MA, USA). The reaction conditions were as follows: pre-denaturation at 95°C for 10 min and 40 cycles of denaturation at 95°C for 15 s and extension at 72°C for 30 s, respectively. U6 was selected as an internal reference of miR-520b, whereas glyceraldehyde-3-phosphate dehydrogenase (GAPDH) was regarded as an internal reference for ZNF367, and the ratio of target genes between the control group and the experiment group was determined based on the 2^−ΔΔCt^ method. The calculation formula: ΔΔCT = Ct_experiment group_ − Ct_control group._^29^ The primers (Shanghai GenePharma, Shanghai, China) used in the experiment are listed in Table 1.

**Table 1:** Primer Sequences of Quantitative Reverse Transcriptase Polymerase Chain Reaction

Gene	Primer Sequence
miR-520b	F: 5′-AAAGTGCTTCCTTTTAGAGGG-3′
	R: 5′-GTGCAGGGTCCGAGGT-3′
U6	F: 5′-GCTTCGGCAGCACATATACTAAAAT-3′
	R: 5′-CGCTTCACGAATTTGCGTGTCAT-3′
ZNF367	F: 5′-AACCGCCACTGTCCGAAGCA-3′
	R: 5′-CCTTTCAAAGTGGGGGTGCGCT-3′
GAPDH	F: 5′-CCACATCGCTCAGACACCAT-3′
	R: 5′-GCGCCCAATACGACCAAAT-3′

miR-520b, microRNA-520b; ZNF367, zinc finger protein 367; GAPDH, glyceraldehyde-3-phosphate dehydrogenase; F, forward; R, reverse.

### Western Blot Analysis

Total protein was extracted from cells in each group, and the concentration of these protein samples was determined using a bicinchoninic acid kit (Thermo Fisher Scientific, Waltham, MA, USA). The total proteins (30 μg) were processed by conducting polyacrylamide gel electrophoresis at 80 V for 35 min and at 120 V for 45 min. Subsequently, the proteins were transformed onto a polyvinylidene fluoride membrane (Amersham Pharmacia, Piscataway, NJ, USA), and 5% skimmed milk was added for conducting membrane blockade for 1 h. Subsequently, the membranes were incubated with the following primary antibodies (Abcam, Cambridge, UK), including rabbit monoclonal antibodies against CD63 (1:1,000, ab134045, Research Resource Identifier [RRID]: AB_2800495), TSG101 (1:1,000, ab125011, RRID: AB_10974262), Ki67 (1:5,000, ab92742, RRID: AB_10562976), and MMP-2 (1:1,000, ab37150, RRID: AB_881512) and rabbit polyclonal antibodies against Alix (1:1,000, ab76608, RRID: AB_2042595), calnexin (1:1,000, ab22595, RRID: AB_2069006), PCNA (1:1,000, ab18197, RRID: AB_444313), MMP-9 (1:1,000, ab73734, RRID: AB_1860201), and β-actin (1:5,000, ab8227, RRID: AB_2305186) overnight at 4°C. The membranes were rinsed using phosphate buffer saline (PBS) Tween 20 (PBST) containing 0.1% Tween 20, 3 times, for 10 min each time. Membranes were incubated for 1 h with the horseradish peroxidase-conjugated goat anti-rabbit secondary antibody (1:1,000; Jackson ImmunoResearch Laboratories, West Grove, PA, USA), followed by 3 PBST rinses (10 min per time). The membranes were visualized using an optical illuminator (General Electric, Boston, MA, USA). The gray-value analysis of the protein bands was performed using Image-Pro Plus 6.0 software (Media Cybernetics, Bethesda, MD, USA).

### 5-Ethynyl-2′-Deoxyuridine (EdU) Staining

The diluted EdU solution (culture medium and EdU at a ratio of 1,000:1) was added to the cell-culture plate for a 2-h incubation at room temperature, followed by a PBS rinse. Next, the cells were fixated using 40 g/L polyoxymethylene for 30 min, incubated in glycine solution for 8 min, and subsequently rinsed using PBS containing 0.5% Triton X-100. Apollo staining solution was added to the samples for a 30-min regimen of incubation at room temperature in conditions devoid of light. Finally, the cells were incubated with Hoechst 3334 culture solution for 20 min at room temperature in conditions devoid of light. The cells were observed under a fluorescence microscope and photographed at an excitation wavelength of 550 nm, and the cells stained in red were reflected as the proliferated cells. The photograph obtained at the 350-nm excitation channel was reflective of blue-stained cells as the total cells. Three visual fields were selected under 400 times, to count the number of EdU-stained cells (proliferated cells) and the Hoechst 33342-stained cells (total cells). Cell-proliferation rate was calculated as proliferated cells/total cells × 100%.

### Transwell Assay

At 48 h post-transfection, cells were starved in serum-free culture medium for 24 h before detachment and then rinsed 2 times using PBS. Afterward, the cells were resuspended using serum-free Opti-MEM I (31985008; Senbeijia Biological Technology, Nanjing, Jiangsu, China) containing 10 g/L bovine serum albumin (BSA) so as to alter the density to 3 × 10^4^ cell/mL. The Transwell chamber was added into the 24-well plates, and the membrane at the basolateral chamber was coated with diluted Matrigel (40111ES08; Yeasen Biological Technology, Shanghai, China) and dried at room temperature. After routine detachment, the plate was rinsed 2 times using PBS, and a cell suspension with cell density of 1 × 10^5^ cell/mL was prepared with the addition of RPMI 1640. Cell suspension (200 μL) was added to the apical chamber, which was coated with Matrigel, and 600 μL RPMI-1640 medium containing 20% FBS was added to the basolateral chamber. After a 24-h routine incubation, the noninvading cells were removed using cotton swabs. Cells invading the bottom of the membrane were fixed using 4% polyoxymethylene for 15 min and stained with 0.5% crystal violet solution for 15 min. An inverted microscope (XDS-800D; Shanghai Caikon Optical Instrument, Shanghai, China) was used for photography and observation. Five visual fields were randomly selected for cell counting. Three duplicate wells were set in each group.

### Flow Cytometric Analyses

Annexin V-fluorescein isothiocyanate (FITC)/propidium iodide (PI) double staining was conducted to detect cell apoptosis. At 48 h post-transfection, the cell density was adjusted to 1 × 10^6^ cell/mL and fixed overnight at 4°C using 70% precooled ethanol solution. A total of 100 μL cell suspension (more than 1 × 10^6^ cell/mL) was centrifuged, resuspended in 200 μL binding buffer, and stained with 10 μL Annexin V-FITC and 5 μL PI in conditions devoid of light at room temperature for 15 min. Eventually, 300 μL binding buffer was added to the cell mixture, and a flow cytometer was applied for assessment of cell apoptosis at an excitation wavelength of 488 nm.

### Exosome Isolation from NFs

NFs were subjected to a regimen of ultracentrifugation at 100,000 *g* for 18 h to remove the exosomes in serum. Upon reaching 80% cell confluence, the supernatant in the culture medium was extracted. Cell suspension was rinsed 2 times with PBS. The NFs were further incubated with exosome-free culture medium containing 10% FBS in a CO_2_ incubator at 37°C for 48 h. The collected supernatant was subjected to centrifugation at 300 *g* at 4°C for 10 min, 2,000 *g* at 4°C, and 5,000 *g* at 4°C for 15 min with removal of the pellets. The collected supernatant was centrifuged at 12,000 *g* at 4°C for 30 min, and the pellet was collected and subsequently centrifuged at 12,000 *g* at 4°C for 30 min. After the differential centrifugation of pellets, the supernatant was extracted and ultracentrifuged at 100,000 *g* for 70 min 4°C. Then, the collected pellet underwent an additional regimen of centrifugation at 100,000 *g* at 4°C for 70 min for collection of the pellet.

### Nanoparticle Tracking Analysis

An amount of 20 μg exosomes was dissolved in 1 mL PBS, oscillated for 1 min to sustain even distribution. Later, a nanoparticle tracking analyzer (NanoSight NS300; Amesbury, Wilkshire, UK) was utilized to measure the size of exosomes.

### TEM Observation

The prepared exosomes were fixated using 4% glutaric dialdehyde at 4°C for 2 h and subsequently fixated using 1% osmium tetroxide for 2 h. Next, the exosomes underwent gradient dehydration with normal ethanol and acetone, followed by infusion, embedding, and polymerization using epoxy resin, and were sliced into 0.5-μm semithin sections for optical mirror positioning. Then, the 60-nm ultrathin sections were stained using uranyl acetate and lead citrate and observed under a TEM microscope (HT7700 Exalens; Beijing SJC Science and Trade, Beijing, China).

### Exosome Transfer into PC Cells

Exosomes (20 μg) were certified to stand at 37°C for 15 min using diluted PKH26 staining solution (1:1,000). The labeled exosomes were rinsed at 100,000 *g* for 70 min. In addition, the cytoskeleton of PC cells was preferentially stained using FITC-conjugated phalloidin (Yeasen Biotechnology, Shanghai, China). Finally, the PKH26-labeled exosomes were cocultured with PC cells for 6 h, 12 h, 24 h, and 36 h, collected at 48 h, resuspended using 500 μL PBS, and stained with 4′,6-diamidino-2-phenylindole (DAPI). The cells were visualized under a confocal fluorescence microscope.

### Detection of Acetylcholinesterase Activity for Exosome Secretion

Exosomes, extracted by performing multistep ultracentrifugation, were diluted using PBS to 110 μL. The diluted exosome suspension (37.5 μL) was plated evenly into each well with 96-well plates, after which, equal amounts of 0.1 mM 5,5′-dithiobis-2-nitrobenzoic acid solution and 1.25 mM acetylthiocholine iodide solution were added into the plate to attain the total well volume of 300 μL. After a 30-min reaction, the plate was observed under a microplate reader so as to measure the optical density value of each well at an excitation wavelength of 412 nm.

### Immunofluorescence Staining

After transfection for 48 h, the cell slide was rinsed 3 times with PBS (5 min each time), fixated using 4% polyoxymethylene at room temperature for 30 min, and rinsed 3 times with PBS again (5 min each time). Then, the section was reacted with 0.2% Triton X-100 at room temperature for 15 min and subjected to a section blockade using 3% BSA at 4°C for 30 min. Subsequently, the cells were incubated with fluorescence primary antibodies against MMP-1 (1:1,000, ab37150; Abcam, Cambridge, UK) and MMP-9 (1:500, ab38898; Abcam, Cambridge, UK) and rinsed 3 times with PBS (5 min each time). Next, the cells were incubated with fluorescence secondary antibody (1:500) at room temperature for 2 h, followed by a PBS rinse. Finally, the cells were stained with DAPI at room temperature in conditions devoid of light for 10 min and sealed using sealing agents for observation under a fluorescence microscope.

### Xenograft Tumor in Nude Mice

Twenty 5-week-old, specific pathogen-free male nude mice, weighing 14∼16 g, bought from Shanghai SLAC Laboratory Animal (Shanghai Laboratory Animal Center of Chinese Academy of Sciences, Shanghai, China) were housed at temperatures of 25°C∼27°C with relatively humidity of 45%∼50%. Ten mice were used for observation of tumor growth at different time points and the remaining 10 mice for observation of tumor metastasis. The involved mice were randomly grouped into the Exo-miR-NSM group and Exo-miR-520b group, with 5 mice in each group, and anesthetized for inoculation. SW1990 cells were cocultured with exosomes isolated from NFs transfected with mimic-NC (Exo-miR-NSM) or miR-520b mimic (Exo-miR-520b). Cells in the logarithmic growth phase following treatment were resuspended using 50% Matrigel (BD Biosciences, Bedford, MA, USA) in order to adjust the density to 2 × 10^6^ cell/mL. A single-cell suspension (4 × 10^5^ cells/0.2 mL) was subcutaneously injected into each mouse via its left axillary vein. On the 7^th^, 14^th^, 21^st^, 28^th^, 35^th^, and 42^nd^ days after instilling the injection, the tumor size of nude mice was measured using a vernier caliper, and the volume of tumor (L stands for the tumor length, and W stands for tumor width) was calculated based on the (L × W^2^)/2 formula. Next, the mice were euthanized, with extraction of liver tissues and division into sections. Finally, H&E staining was performed to count the number of lymph metastatic nodes.

### Statistical Analysis

All data were analyzed using SPSS 21.0 software (IBM, Armonk, NY, USA). Measurement data were expressed as mean ± standard deviation. Independent-sample t test with Welch’s correction was adopted for comparison between two groups. Shapiro-Wilk test was performed for testing normality of data among multiple groups. Comparisons of data obeying normal distribution among multiple groups were analyzed with one-way analysis of variance (ANOVA). Moreover, the least significant difference test was applied for pairwise comparison among multiple groups. Nonparametric Kruskal-Wallis test was performed for comparisons between data, not conforming to normal distribution. A value of p < 0.05 was considered to be statistically significant.

## Author Contributions

H.S. designed and performed the study, analyzed the data, and wrote the manuscript. X.Z. and H.L. designed the study. T.Z. and Y.D. collated the data, carried out data analyses, and produced the initial draft of the manuscript. X.P. and H.S. contributed to drafting the manuscript. All authors read and approved the final manuscript.

## Conflicts of Interest

The authors declare no competing interests.

## Supplemental Information

Document S1. Figure S1

Document S2. Article plus Supplemental Information
